This article has been retracted.

# Femtosecond Laser Combined with Double-Flange Polypropylene Suture Capsular Tension Ring Suspension for the Treatment of Subluxation of Lens in Marfan Syndrome

**DOI:** 10.1155/2022/9348311

**Published:** 2022-08-10

**Authors:** Li Zhou, Shangcao Wu, Huafang Guo

**Affiliations:** Ophthalmology Department, Aier Eye Hospital of Wuhan University, Wuhan, China 430066

## Abstract

**Purpose:**

To evaluate the use of femtosecond laser combined with double-flange polypropylene suture capsular tension ring (CTR) suspension to treat subluxation of lens in Marfan syndrome. The objective is to provide safer and more effective surgical procedures for patients. S*etting*. Eye Hospital, Aier Eye Hospital of Wuhan University, Wuhan, China

**Methods:**

In this retrospective study, we observed sixteen patients (16 eyes) with Marfan syndrome who had undergone this operation. Femtosecond laser incision was performed on the anterior capsule with the lens as the center. The suspending CTR was clipped to anterior capsule to support it, which was secured to the sclera with a double-flange polypropylene suture. Uncorrected visual acuity (UCVA), intraocular pressure (IOP), tilt, and decentration of the intraocular lens (IOL) and postoperative complications were evaluated.

**Results:**

All 16 patients were successfully implanted with suspended CTR and IOL after femtosecond laser assisted surgery. Visual acuity improved significantly after surgery (*p* < 0.01). At 1 month, 3 months and 6 months postoperatively, the tilt of the IOL was 2.70 ± 0.934, 2.65 ± 0.897, and 2.66 ± 0.781, and the decentration of the IOL was 0.30 ± 0.770, 0.30 ± 0.682, and 0.29 ± 0.737; both had no statistically significant difference between the three groups. After the operation, 4 patients had hyphema and 2 patients experienced a temporary postoperative IOP increase. Only one flange was exposed one month after operation and recovered right after secondary adjustment.

**Conclusion:**

Femtosecond laser combined with double-flange polypropylene suture CTR suspension was effective in fixing the lens capsule to the scleral wall in cases of subluxation of lens seen in Marfan syndrome during our short-term observation. The long-term efficacy of this operation needs further observation and follow-up.

## 1. Introduction

Marfan syndrome (MFS) is an irregular chromosomal dominant disease with clinical phenotype that involves multiple systems throughout the body, with an incidence of 0.02%~0.01%, generally more males than females [1]. Marfan syndrome was first reported in 1896 [2]. The clinical manifestations of Marfan syndrome are diverse due to multisystem congenital dysplasia. The main lesions can be accumulated in the cardiovascular system, skeletal system, eye system, respiratory system, and skin system [3]. The ocular signs are retinal detachment, refractive error, nystagmus, glaucoma, strabismus, amblyopia, and lens ectopic. Both the lens subluxation and dislocation are also its typical clinical manifestations of eye, incidence of about 60%, whereby the ectopic lens will seriously affect the development of visual function; and if not treated, it will cause visual impairment therefore affecting the patients' quality of life [4]. In recent years, with the improvement of surgical techniques and the progress of surgical equipment, personalized surgical plans for patients having lens subluxation are also constantly improved while hoping to provide a better guarantee for the maximum recovery of patients' visual function.

Incomplete dislocation of the lens had previously been a contraindication for phacoemulsification. The traditional treatment method is to remove the dislocated lens intracapsular or extracapsular and fix the posterior chamber Intraocular lens (IOL) with scleral sutures or implant anterior chamber IOL [5]. With the development of science and technology, phacoemulsification has developed rapidly. Capsular tension ring (CTR) is a milestone in lens subluxation surgery, which enables intracapsular implantation of IOL to position the IOL in a physiological position and achieve better visual effects [6, 7]. Part of the patients with CTR implantation can still have the dislocation of the CTR-IOL capsular complex, so for patients with severe lens incomplete dislocation, the use of simple CTR implantation is unstable [8]. Suspending CTR can fix the capsular bag and make it possible to implant the IOL into the capsular bag. The capsulorhexis is one of the most difficult steps of phacoemulsification in the surgical treatment of lens subluxation. Competence in this area is critical to safe and efficient cataract surgery [9]. Chen et al. believe that femtosecond laser (FL) combined with suspending CTR implantation is an ideal approach to the treatment of traumatic lens dislocation [10]; though suspending CTR are fixed in the scleral surface sutures, intraoperative sutures were crossed back and forth into the sclera; it still has the conjunctiva incision therefore making the postoperative suture irritation unavoidable. We used femtosecond laser combined with double-flange polypropylene suture CTR suspension to treat subluxation of lens in Marfan syndrome, since it makes the operation easier and more convenient. The report is as follows:

## 2. Objects and Methods

### 2.1. Objects

16 eyes of 16 Marfan syndrome patients with subluxation of lens were collected from January 2018 to December 2020 in Aier Eye Hospital of Wuhan University, including 12 males and 4 females. The age ranged from 18 to 37 (average 24.38 ± 4.965) years. The dislocation range is 90°to 180°. Preoperatively, corrected visual acuity of 11 eyes were less than 0.3 and 5 eyes had a visual acuity of less than 0.1, no anterior chamber vitreous prolapse and secondary glaucoma, and no aortic dissection.

### 2.2. Method

#### 2.2.1. Preoperative Examination

All patients underwent uncorrected and corrected vision, natural pupil, dilated slit lamp examination, ultrasound biomicroscopy (UBM), intraocular pressure (IOP), IOLmaster 700, Optical Coherence Tomography (OCT), and fundus examination before operation.

#### 2.2.2. Surgical Method

The pretreatment was performed with the LenSx laser (Alcon Laboratories, Fort Worth, TX, USA). After successful docking of the laser-patient interface, spectral domain optical coherence tomography (OCT) imaging of the anterior segment was performed. Images of the intraocular structures were automatically identified. The surgeon confirmed each step of the procedure in accordance with the necessary safety margins. After that, the laser treatment was initiated and included creating a 5.2 mm capsulotomy with the lens as the center, capsule delta up and down both 350 *μ*m (Figure 1). Once the FL pretreatment was completed, phacoemulsification was performed using the Centurion Vision System (Alcon Laboratories).

Clear corneal primary and lateral incisions were made; the dispersive ophthalmic viscosurgical device (OVD) (Viscoat, Alcon Laboratories) was injected into the anterior chamber to protect the endothelium. The anterior capsule was removed with capsulorhexis forceps. One or 2 capsular hooks were placed on the side of the lens dislocation according to the rupture scope of the suspensory ligament to stabilize the lens capsular bag. The other end of the 7-0 polypropylene suture with one end made into a flange was passed through the suspension hole of the tension ring; also, the tension ring of the pre-set suture was implanted into the capsular bag and adjusted so that the suspension hole was located in the middle position of the lens dislocation. The 30-gauge needle punctured the bulbar conjunctiva from the 2 mm scleral surface behind the corneal limbus and entered the eyeball after walking a tunnel through the sclera. The posterior surface of the iris was carefully closed; we pulled the other 7-0 polypropylene suture thread out. The cataract surgery was then completed with standard phacoemulsification procedure with a phaco-and-chop technique. The remaining cortex was removed with coaxial irrigation/aspiration. Cohesive OVD (Provisc, Alcon Laboratories) was injected to expand the anterior chamber and capsular bag, followed by intraocular lens (IOL) implantation. Visco in the anterior chamber and after the IOL was removed. 7-0 suture was tightened until the bag was centered. The outer end of the suture was cut short and heated to make a flange as well as riveted on the sclera surface (Figures 2 and 3). Then, the pupil was dilated with carbacholine. At the end of the procedure, stromal hydration was applied to close the corneal incisions. A combination steroid-antibiotic ointment was therefore placed on the eye in addition to covering the eye with a patch.

#### 2.2.3. Follow-Up Postoperative

The patients were followed up for 6 months. UCVA, position of the postoperative capsular complex, hemorrhage, IOP, and flange exposure were recorded.

## 3. Results

All 16 patients were successfully implanted with suspended CTR and IOL. There were no serious surgical complications during the operation, such as massive intraocular hemorrhage and rupture of the capsular bag. In 4 patients, the 30-gauge needle touched the iris, causing a small amount of intraocular bleeding. After cutting the vitreous body located in the incision and pupil area, the pupil was round and the incision was watertight. After surgery, elevated IOP was observed in 2 patients on the second day. All recovered normally one week after surgery. Only one flanges was exposed one month after the operation and recovered after secondary adjustment (Table 1). Afterwards, the visual acuity was improved in comparison to that before the operation (*p* < 0.01) (Table 2). At 1 month and 3 months to 6 months postoperatively, the tilt of the IOL was 2.70 ± 0.934, 2.65 ± 0.897, and 2.66 ± 0.781, and the decentration of the IOL was 0.30 ± 0.770, 0.30 ± 0.682, and 0.29 ± 0.737; both had no statistically significant difference between the three time points (Table 3). There was no obvious tilt or decentration of the IOL in postoperative follow-up.

## 4. Discussion

The core of modern surgical treatment for incomplete lens dislocation is to maximize the retention and remodeling of the lens capsular suspensory ligament septum [11–14], which can reduce the harassment of vitreum and the occurrence of posterior segment complications. A complete and suitable continuous circular capsulorhexis is also a prerequisite. In the case of lens dislocation, due to the weakening of the suspensory ligament resistance, manual capsulorhexis becomes difficult.

FL capsulorhexis is the biggest highlight of femtosecond laser-assisted cataract surgery. It has unique advantages in complex cases such as cataracts with unstable zonules and partial separation [15, 16]. In cases of lens dislocation, FL anterior capsule incision should be set with the lens as the center, rather than the pupil as the center to ensure the neutral position of the anterior capsule opening and the incision diameter should not be too large. In addition, during operation when the patient lies flat, the lens is tilted backward. At this time, the position of the anterior capsule at the dislocation site is low which may lead to incomplete laser cutting. In order to ensure that the anterior capsule of the dislocation is within the incision range, the lowest point of femtosecond laser incision at the dislocation can be accurately located under real-time OCT scanning. In this study, 16 patients underwent FL capsulorhexis with no incomplete capsulorhexis and no capsular rupture occurred.

The CTR is a promising option for patients with ectopia lentis who require lensectomy. Inserted into the capsular bag, this device has provided both intraoperative and postoperative stabilizations of the capsular bag-IOL complex. The standard CTR is an open, compressible ring of polymethylmethacrylate with a single eyelet at each end [17, 18]. By providing centrifugal force at the capsular equator distributed equally around the zonular apparatus, the CTR stabilizes weak zonules by recruiting stronger ones [19–21]. It also decreases the occurrence of postoperative capsular traction and posterior capsular opacification formation. For either of these conditions, it is not adequate to recenter a severely subluxed lens or preventing progressive zonular loss. But we may consider a modified CTR, which may be sutured to the scleral wall because capsular tears may be the result from suturing the CTR through the capsular bag. The modified CTR was designed to address this complication [22]. The modified CTR has one or two fixation eyelets that protrude 0.25 mm anteriorly from the ring; once the modified CTR is in place, these eyelets sit anterior to the anterior capsule and provide an anchor for sutures while allowing for uncompromised integrity of the capsule itself [23]. Typically, the eyelets are sutured in the direction of zonular weakness.

In patients with Marfan syndrome, the lesion of suspensory ligament of the lens is progressive, and the lesion range is often more than one quadrant. However, the standard CTR has no fixed hook of suture, so its long-term clinical effect is not good after implantation. Therefore, we recommend the use of modified CTR in the treatment of Marfan syndrome patients with lens dislocation. Based on the traditional standard tension ring design, it adds one or two suturing handles with fixed rings at the top in the middle of the ring, which can not only expand the pressure of the bag as well as keep the bag round but also fix the bag by suturing which is conducive to maintaining the long-term stability of the bag and the neutral position of the IOL [24, 25]. At the same time, it can resist the shift of pouch tension ring caused by lens epithelial cell proliferation and migration to a certain extent making it more suitable for young Marfan syndrome patients.

The timing of the suspension CTR implantation is more important. Usually, the lens nucleus of patients with traumatic lens dislocation is relatively soft. CTR can be implanted after phacoemulsification or coaxial irrigation/aspiration if the surgery is expected to be easier, CTR is recommended to be implanted after capsulorhexis or hydrodissection [26, 27]. Wulin et al. compared the surgical effects of first-stage implantation of modified CTR and scleral fixation, or first-stage implantation of CTR, and the second-stage CTR-capsular composite scleral fixation after 3-6 months. Xinyan et al. used phacoemulsification-combined suspension CTR implantation [28]. Both successfully retained the capsular bag and implanted the posterior chamber IOL.

Therefore, for a wide range of lens dislocations, the suspension CTR is helpful to the safety of surgery and shows excellent application prospects [29, 30]. It broadens the scope of application of posterior chamber IOL implantation. However, most surgeons sew sutures under the scleral flaps and on the surface of the conjunctiva therefore making the operation more complicated also causing obvious suture irritation after operation [31–33].

The characteristic of this study is the 30-gauge needle used to enter the anterior chamber after a scleral tunnel; the puncture port is closed without suture, so there is no need to make scleral flap and cut the bulbar conjunctiva. The broken end of the 7-0 polypropylene thread exposed outside the eyeball is processed into a flange at high temperature and riveted on the scleral surface instead of the traditional knotting to reduce the suture stimulation. Not only does it shorten the operation time but also minimizes the damage to the eyeball tissue. Moreover, the flange is similar to a disc, so it is not easy to be exposed to the ocular surface due to puncturing the bulbar conjunctiva. The 16 patients in this study had no discomfort after 6 months of follow-up including suture stimulation, suture exposure, and flange slippage. The 7-0 polypropylene thread had a larger diameter than the 10-0 polypropylene suspension thread, so the IOL-capsule complex was not easy to fall off. Studies have reported that the suspension line of the suspension CTR can only be passed through the protruding suspension ring and the position of the suspension ring must be aligned, well-adjusted to an accurate position in order to suture successfully [34–37]. Cai and Lele believe that the suspension ring protruding above the capsular bag also increases the risk of friction with the iris [38–41]. So they used ordinary CTR for tension ring suspension. However, when using ordinary CTR for suspension, the needle has to pass through the lens capsule, risking tearing of the capsular bag. There is no such worry about using the suspended CTR. Only one case of flange exposure occurred one month after operation and recovered after secondary adjustment in this study. We considered that due to the friction between flange and conjunctiva, it is necessary to accumulate more cases and follow-up for a longer time. In addition, when the range of lens dislocation is too large, the capsular bag should not be retained, and the stability of the postoperative CTR-capsular bag complex should be comprehensively evaluated.

## Figures and Tables

**Figure 1:** The pretreatment was performed with the LenSx laser; the parameter setting included creating a 5.2 mm capsulotomy with the lens as the center, capsule delta up and down both 350 *μ*m. (A) The arrow displays the capsulotomy parameter setting. (B) The arrow displays the capsule delta up and down parameter setting.

**Figure 2:** The suspending CTR was implanted into to anterior capsule to support it, which was secured to the sclera with a double-flange polypropylene suture. The blue line segment in (a) describes the alignment of the double flanges.

**Figure 3:** The photograph of the subconjunctival flange 6 months after surgery. The arrow displays the stage of the flange.

**Table 1:** Patient characteristics and complications at 1 day postoperatively (POD1) and 1 month postoperatively (POM1).

	Eyes (*N* = 16)	
	Number	(%)
Gender		
Male no. of eyes (%)	12	75%
Female no. of eyes (%)	4	25%
Average age (years)	24.38 ± 4.965	
Postoperative complications		
Hyphema (POD1)	4	25%
Elevated IOP (POD1)	2	12.5%
Flange exposure (POM1)	1	6.25%

**Table 2:** The UCVA before and after operation was compared.

	Preoperative	POD1	POD1	POM1
UCVA	0.075 ± 0.533	0.461 ± 0.274	0.461 ± 0.274	0.638 ± 0.175
*t*	-5.544		-2.172	
*p*	<0.01		0.038	

**Table 3:** The IOL tilt and IOL decentration after POM1, POM3, and POM6 were compared.

	POM1	POM3	POM6	*t* ^a^	*p* ^a^ (POM1 vs. POM3	*t* ^b^	*p* ^b^ (POM1 vs. POM6)
IOL tilt	2.7 ± 0.934	2.65 ± 0.897	2.66 ± 0.781	0.154	0.878	0.21	0.983
IOL decentration	0.3 ± 0.770	0.3 ± 0.682	0.29 ± 0.737	-0.049	0.96	-0.448	0.657

POM1: 1 month postoperatively; POM3: 3 months postoperatively; POM6: 6 months postoperatively. ^a^Between postoperative 1 month and 3 months. ^b^Between postoperative 3 month and 6 months.

## Data Availability

The data in this study are all from Aier Eye Hospital, which is real and effective.
